The article "Green investing in China's air cargo industry: Opportunities and challenges for sustainable transportation" was retracted in 2025. Reasons: unreliable results or conclusions; concerns about the citations.

# Green investing in China's air cargo industry: Opportunities and challenges for sustainable transportation

**DOI:** 10.1016/j.heliyon.2023.e19013

**Published:** 2023-08-08

**Authors:** Weisong Wang, Wenjing Sun, Usama Awan, Abdelmohsen A. Nassani, Rima H. Binsaeed, Khalid Zaman

**Affiliations:** a School of Marxism, Xinjiang Normal University, WuLuMuQi 830017, China; b School of Marxism, Guangxi Science and Technology Normal University, LaiBin 546199, China; c Center for Research on Digitalization and Sustainability, Inland Norway University of Applied Sciences, Norway; d Department of Management, College of Business Administration, King Saud University, P.O. Box 71115, Riyadh, 11587, Saudi Arabia; e Department of Economics, The University of Haripur, Haripur Khyber Pakhtunkhwa 22620, Pakistan

**Keywords:** Air cargo operations, Carbon damages, Transportation fuel combustions, Greenfield investment, Insurance services, China

## Abstract

Aviation cargo remains vital in the economic activities to transported goods from one place to another. The developed and developing countries mainly consider the transaction routes for air transportation for safe and quickest mode. Chinese economy is attracting the global World through its exports. The country's air cargo system is mainly reliant on gasoline and petroleum-based fuels, which harms the country's green transportation agenda. The high use of fuel combustions in the aviation sector needed greenfield investment that helps to use green energy as an alternative sustainable fuel. Further, sustainable aviation insurance and financial coverage are needed to mitigate the adverse negative externalities from air cargo operations. Based on the crucial facts, the study used air cargo operations, transportation fuel combustions, private investment in the transportation and insurance coverage in the pollution damage function for the China economy using data from 1975 to 2020. The research employed a non-linear ARDL Bounds testing strategy to break down the sequence of variables into dynamic positive and negative multipliers. Positive shocks in air freight, insurance services, and greenfield investment have been shown to reduce carbon emissions immediately and over the long term. In the short term, carbon damages are exacerbated by the negative shocks resulting from the use of transportation fuel and the availability of insurance. Moreover, both the positive and negative shocks associated with transportation fuel combustions and air transportation freights contribute to a rise in carbon damage. The variance decomposition analysis validated the asymmetric correlations between the aforementioned variables in the intertemporal environment. Based on the findings, negative shocks from total fuel combustions are expected to impose the greatest carbon damages over the next decade, followed by insurance services and air freight operations. The study concludes that air cargo operations need to be sustainable transacting routes fueled by biofuel energy sources, greenfield investment, and sustainable aviation insurance coverage to achieve the ‘green is clean’ transportation agenda.

## 1 Introduction

The multimodal transportation routes are mainly used for cargo operations worldwide. Air cargo, roads, rail, and water use for goods shipped from one place to another [1]. Numerous airports and airlines, both inside China and abroad, provide China with one of the world's most comprehensive air freight networks [2]. Shanghai Pudong, Beijing Capital, and Guangzhou Baiyun International Airport are three of China's most crucial cargo airports. These airports process a great deal of cargo and are major local and international shipping hubs [3]. Several Chinese airlines focus only on shipping goods by air. China Cargo Airlines, SF Airlines, and Cathay Pacific Cargo are all significant participants in the cargo airline industry [4]. Freighters like the Boeing 747, Boeing 777, and Airbus A330 are just some of the planes these carriers fly. Cargo services provided by passenger airlines use the aircraft's belly room to convey goods by air. Due to jet fuel combustion, air freight activities are linked to substantial amounts of carbon emissions. About 2.8% of the world's human-made carbon emissions came from aviation in 2019. Cargo aircraft account for a lesser share of these emissions than passenger flights, but they have a significant impact on global carbon production. In 2021, major Chinese airlines transported 7.3 million metric tons of goods and mail via air. China has recognized the need to reduce carbon impacts and increase sustainability in the aviation industry because of the environmental effect of air freight operations [5]. One such step is encouraging fuel-efficient planes like the Boeing 787 and Airbus A350, which use less fuel per ton of cargo delivered. Spreading awareness of SAF, which, compared to regular jet fuel, may cut carbon emissions by as much as 80%. China has been heavily investigating and investing in SAF manufacturing and use. Spending money on infrastructure to support electric and hybrid-electric freight planes to cut down on future fossil fuel use. Decrease fuel use and emissions by implementing state-of-the-art air traffic management technologies, optimizing flight paths, and reducing congestion. China's economic development and international commerce depend critically on its air freight operations. However, the carbon harms caused by these activities must be addressed immediately [6]. China plans to lessen the negative impact of its air freight operations on the environment via eco-friendly policies, cutting-edge technology, and initiatives, including sustainable aviation fuels. Maintaining a sustainable economy while minimizing the carbon footprint will need ongoing work [7,8].

According to the Carbon Brief [9] report, China is one of the leading aviation emissions countries to increase four times higher carbon emissions by 2050. The World Bank [10] database shows that the Chinese economy faces higher carbon damages to 7.024% of GNI in 1995, latter decreases to 6.036% in the year 2005. Further, approximately half of the carbon damages decreased and reached the level of 3.201% in 2015 and 3.086% in 2020. Besides many economic and environmental factors, air cargo operations consider a vital factor that adversely affects the country's air quality level. A substantial increase in aviation cargo operations was observed from 46.2 million ton-km in 1975 to 403 million ton-km in 1985. This figure increases many times during the analysis of the country's decade data set, further increases from 1501 million ton-km to 7579 million ton-km in the subsequent two decades (i.e., 1995's and 2005's decades). Moreover, air transportation freight increases to their maximum level in 2020 with a number count of 25394 million ton-km. The higher carbon-induced transportation fuel combustions get a peak value after 2005 from 7.710% of total fuel combustions to 8.599% in the current year. The greenfield investment in the transportation sector shows a lacuna in a country-centric policy related to the green developmental process. The private participation in transportation investment substantially declines from the year 2005 to 2020 with a US$ 6,628,900,000 to US$2,788,890,000. Among many possible reasons, one crucial factor is that the country's insurance and financial services decrease from 1995 to 2020 by 16.942% to 4.114%, respectively. The given statistics confirmed the unsustainability in the air cargo operations, leading to carbon damages. It had many different factors, including non-renewable kerosene fossil fuel used in aviation cargo operations, low green field transportation investment, and meager insurance and financial services in a country. Financial support is a crucial component in ensuring the smooth operation of economic activities [11]. Succession planning and strategic investments help to move forwards towards economic prosperity [12,13]. Fig. 1 shows the trend analysis of the stated factors for ready reference.

**Fig. 1:** Data trends of air cargo operations and carbon damages in China.

Source: World Bank [10].

Given its importance in China's economic activity and its influence on carbon emissions, this research focused on its air freight business. While marine transport accounts for a significant portion of world emissions, various reasons led to examining the air freight sector [14]. The first is that air freight is essential for delivering time-sensitive and high-value commodities because of the speed and security it provides during transit. Because of China's growing exports and status as a worldwide trading center, the air cargo business is significant to analyze for its ecological footprint. Although marine transport is anticipated to contribute significantly to future emissions, it is essential to recognize that each mode of transportation has distinct features and problems regarding reducing emissions. This research set out to investigate the environmental effects of the air freight business and provide suggestions for reducing carbon emissions in this sector.

Previous studies have offered various sustainable solutions to enhance air cargo operations, linking them to the study's first hypothesis. These solutions include bioenergy consumption [15] and the deployment of alternative-energy vehicles [16]. Other solutions include sustainable technical innovation in transportation [17] and developing an efficient energy system [18,19]. In addition, the second hypothesis of the study is in line with previous research that has emphasized the importance of creating a private partnership investment opportunity in the transportation sector to advance the green transportation agenda [[20], [21], [22], [23], [24]]. Finally, the following investigations lend credence to the third hypothesis [[25], [26], [27]]. This research advocates sustainable insurance coverage to reduce economic and transportation losses. The study needs to answer the following research questions, i.e., does unsustainable cargo operations increase the cost of carbon pollution in a country? The question stressed the need to improve cargo operations through low carbon travelling mode to reduce energy demand and achieve energy efficiency. The second question is: to what extent do adverse environmental externalities arise due to transportation fuel combustion? The question argued that unsustainable aviation fuels harm the green transportation agenda, which can improve by using biofuels in aviation to perform their logistics operations. Finally, does greenfield investment in transportation improves aviation performance to reduce carbon pollution? The private investors remain curious to improve aviation performance through running sustainable logistics operations. Hence, the green investment covered by sustainable insurance schemes helps attain the stated green agenda to improve the transportation system. The study's research objectives have set in line with the research questions, which are as follows:

i) To examine the impact of aviation cargo performance on carbon damages in a country.
ii) To investigate the role of greenfield investment in the transportation sector in mitigating carbon pollution, and
iii) To evaluate the impact of transportation fuel combustion and insurance & financial services in pollution damage function.

These objectives, along with the research questions, need to be checked by different time-varying statistical techniques that help get the deviation in the stated factors on the outcome variable during the stated period.

## 2 Literature review

There is a wealth of research on air travel, economic development, and environmental costs in various economies. An index measuring the relative attractiveness of 19 countries as tourist destinations were created by Khan et al. [28]. They spoke about how international travel by plane and train affects domestic and international tourism. The findings backed up the practicality of various modes of transportation and tourist destinations on the global stage. Air and rail transportation was shown to have bidirectional causal implications concerning international tourist infrastructure. The research found that a country's ability to provide secure and convenient access to several modes of transportation was a significant factor in luring visitors from outside. Using data from 1990 to 2015, Nassani et al. [29] analyzed the impact of railroads on fossil fuel energy consumption, N2O, and GHG emissions across BRICS nations. According to the findings, there is a significant rise in the need for fossil fuel burning, N2O emissions, and GHG emissions associated with travel and transport services and the shipment of commodities by railroads. Nonetheless, carbon pricing and renewable energy sources are beneficial in reducing the global effect of emissions. In order to realize a green transportation agenda, transportation infrastructure must be constantly upgraded. The utilization of green energy is crucial to the BRICS countries' goal of carbon neutrality. The connections between air and rail transportation and environmental deterioration were examined by Saleem et al. [30] in a panel study of 11 nations spanning 1975–2015. The findings indicate that transportation considerations and energy consumption negatively impact the natural environment and resource capital. The global price of carbon pollution may be lowered by implementing green transportation legislation and bilateral funding. Improve air quality indicators and protect Pakistan's natural resource capital by investing in green transportation infrastructure, as Shouket et al. [31] emphasized. Transportation improvements, sustained economic expansion, and the diffusion of cutting-edge technologies are necessary to achieve the desired future state. To investigate the impact of air cargo operations on greenhouse gas emissions, Anser et al. [32] collected data on the Arab world as a whole from 1975 to 2018. The findings suggested a connection between air cargo operations and rising carbon footprints caused by unsustainable fuelling in freight processes. However, uncontrolled environmental variables, such as unsustainable inward Investment supporting the ‘pollution haven’ argument, render carbon price ineffective at reducing carbon footprints. The primary goal is to achieve a carbon-neutral freight business by switching from traditional kerosene to biofuel.

The logistics operations should be green and clean to support the global supply chain process. The sustainable logistics procedure helps to decrease energy demand and achieving energy efficiency through technology spillovers. Carbon taxes can mitigate carbon footprints through cargo operations [[33], [34], [35]]. The current strike of literature available on transportation services and environmental considerations embeds the need for sustainable transportation operations to improve air quality levels. Chen et al. [36] argued that high-speed rail has a minimal effect of carbon offset in Beijing, China, because the traffic volume was unprecedentedly high due to the diversion of air-railways passengers to the high-speed rail. Thus, it turns to negatively impact on environmental quality in the form of escalating carbon emissions. Yuan et al. [37] proposed restricting international tourists at a certain level of visitations allowed in the destination place to control carbon footprints. Pricing theory is the best policy option to limit carbon emissions in tourist's destinations. Sohail et al. [38] found an asymmetric relationship between air-railways transportation and carbon emissions in Pakistan by using data from 1991 to 2009. The positive and negative shocks of transportation confirmed the volatility in the sustainable policy mix that need to be balanced through improving green transportation infrastructure. Godil et al. [39] emphasized the need to adopt green energy fueling in the transportation sector to reduce ecological footprints. Further, it is necessary to attract foreign investors to produce eco-friendly goods to help attain a green developmental agenda. Shafique et al. [40] found that transportation infrastructure is not capable enough to mitigate adverse environmental externalities in a panel of 10 Asian countries. Hence, it is desirable to propose different sustainable policy options to help build green transportation infrastructure across countries.

Fang [41] examines the connection between financial complexity, power industry ventures, green technology innovation, and the layout of industries. The study concludes that the rising trend in carbon emissions may be attributed to the financial complexity measure. In contrast, investments in energy efficiency, ecological technology, and business structure may lower emissions. The study concludes with policy suggestions in light of these results. Liu and Yuan [42] use the United Nations indicator framework to analyze 11 transport indicators to understand better China's progress toward a more sustainable transportation system. The study praises China's transportation system and points out its weaknesses in clean power utilization and uneven bus ownership across regions. The wavy character of China's progress toward a more sustainable transport system is shown by examining indicators' interactions and spatial patterns. In the wake of the pandemic, Zhao et al. [43] investigated the idea of green economic recovery (GER), stressing the need to balance the two goals. In order to achieve sustainable development in the post-epidemic age, this study reviews the literature and GER policies in China and worldwide. The findings aid in clarifying the advantages and disadvantages of various green recovery strategies. Chen et al. [44] examine China's transportation sector's carbon emissions and decoupling progress. The research suggests a unified analytical strategy and pinpoints investment and carbon intensity as significant contributors to GHG production. It shows that decoupling trends are modest and that transitions to decoupling vary among regions. Insights into low-carbon growth in the transportation industry are presented, together with possible future scenarios for carbon emissions and decoupling. The effects of clean power technology and digital finance on green development in China's provinces are investigated by Razzaq et al. [45]. The results show that although both central and eastern areas benefit from digital finance's promotion of green development, the East benefits more from cleaner technology than the latter. The study shows that regional differences and government action are crucial for green development.

Based on the substantial discussion, the study proposed the following research hypotheses, i.e.,

H1 Air cargo operations are likely to increase carbon damages because of fossil fuel combustions in transportation.

H2 Greenfield investment in the transportation sector would likely exert a positive impact on environmental quality, and

H3 Sustainable insurance and financial services are likely to decrease carbon damages in a country.

The study contributed to the existing studies into three main aspects. First, the study used an asymmetric relationship between air cargo and carbon damages in the context of China, while the previous studies mainly concise their findings on the symmetric relationships between them [[46], [47], [48], [49]]. The asymmetry in the modelling framework would likely give more pragmatic solutions to the policymakers to devise green transportation policies to improve aviation performance. Second, the study used greenfield investment in transportation as a potential regressor of the carbon damage function, which inbound FDI previously fills. The greenfield investment allows private investors to play an influential role in mitigating carbon pollution. Hence, foreign investors always try to get sustainable policy solutions to improve the transportation sector [[50], [51], [52], [53]]. Third, the transportation fuel combustion included in the pollution damage function harms the green aviation agenda. The earlier studies mainly limited their findings to suggest substituting gasoline and petroleum-based fuels with biofuels. At the same time, they overlooked to subsidize it through sustainable insurance & financial coverage to improve aviation performance [[54], [55], [56], [57], [58]].

## 3 Data source and methodological framework

The study investigated the asymmetric relationship between air cargo and carbon damages, controlling transportation fuel combustion, greenfield investment, and insurance services in the context of China by using data from 1975 to 2020. Carbon damages (denoted by CDAM, % of GNI) serve as the outcome variable. The remaining variables, including air transportation freight (denoted by ATF, million ton-km), transportation fuel combustion (denoted by TFC, % of total fuel combustion), greenfield investment in transportation (denoted by GFIT, current US$), and insurance and financial services (denoted by IFS, % of service imports) served the predictors variables. The data series of TFC is missing for the year 2015 onward. The GFIT data is available from 1990 onward, and IFS data is missing from 1975 to 1981. The study does not self-generate the missing values while it is filled from the preceding and succeeding values of the same variable to avoid any variations. The data of the candidate variables were collected from the World Bank [10].

China used a multimodal transportation system for cargo goods from one place to another. Air cargo use for safe and quickest shipment. Gasoline, petroleum and other transportation fuels use for this purpose. The country's economic growth is fueled by the larger transactions of their goods to exports abroad. However, the country bears carbon emissions due to unsustainable shipments that damage the green developmental agenda. The public-private investment in the transportation sectors is helpful to find new avenues of sustainable transportation and cargo system linked it with the insurance coverage to minimize carbon damages in a country. The study offered the ‘green transportation theory’ where air cargo and aviation fuels influenced the natural environment, causing greater environmental damages due to unsustainable transportation systems. The use of biofuels in the aviation sector is helpful to reduce carbon damages, which required greenfield investment and insurance coverage to improve air quality levels. Fig. 2 shows the suggested mechanism of adopting green transportation in a country.

**Fig. 2:** Green transportation system.

Source: Adapted from Li [59], Yilmaz &Atmanli [60], and Sivoplyasova & Voinov [61].

Based on the theoretical importance of the stated factors, the study used the following equation (1) to analyze the green transportation system in a country, i.e.,

(1) $$\begin{array}{l} CDAM=\alpha_{0}+\alpha_{1}ATF+\alpha_{2}TFC+\alpha_{3}GFIT+\alpha_{4}IFS+\varepsilon \end{array}$$

Where CDAM shows carbon damages, ATF shows air transportation freight, TFC shows transportation fuel combustion, IFS show insurance & financial services, and ε shows error term.

Equation (1) shows that air cargo activities and aviation fuel combustions can check a green transportation system that increases carbon damages. Further, private investment in the transportation sector to become fuel efficient and insurance coverage helpful to mitigate adverse environmental concerns to achieve sustainable development agenda. Equation (1) is the general specification of the estimated model that can be written in the non-linear ARDL (NARDL) specifications. The NARDL technique absorbed both the positive and negative shocks of the stated factors to check the asymmetry plots in the candidate variables. It estimated the short- and long-run parameter estimates. The study decomposed three potential regressors based on their viability of the dynamics obtained in the estimation to capture positive (+) and negative (−) shocks that yield six different outcomes. Zaman [62] expanded the application of the ARDL approach to include cross-panel data sets.

The NARDL Bounds testing technique is similar in many aspects of the conventional ARDL bounds testing approach proposed by Pesaran et al. [63]. However, the main difference is to generate positive and negative asymmetry plots in the candidate variables, which can yield different outcomes. For similarity aspects, the NARDL is equally applicable for the small sample size, can be used for either level variables or first differenced variables, or mixed order of integration, except second difference operators, and generate short- and long-run parameter estimates. The simple asymmetric cointegrating equation (2) can use for NARDL specification, i.e.,

(2) $$CDAM_{t}=\delta_{0}+\delta_{1}ATF_{t}^{+}+\delta_{2}ATF_{t}^{-}+\delta_{3}TFC_{t}^{+}+\delta_{4}TFC_{t}^{-}+\delta_{5}GFIT_{t}+\delta_{6}IFS_{t}^{+}+\delta_{7}IFS_{t}^{-}+\varepsilon_{t}$$

Where CDAM shows carbon damages, ATF^+^ and ATF^−^ shows positive and negative shocks in air transportation freight, TFC^+^ and TFC^−^ shows positive and negative shocks in transportation fuel combustion, GFIT shows greenfield investment in transportation, and IFS^+^ and IFS^−^ shows positive and negative insurance & financial services, and ε shows error term.

Equation (3) shows the NARDL specifications, i.e.,

(3) $$\Delta CDAM_{t}=\eta_{0}+\sum_{k=0}^{p}\eta_{1}\Delta CDAM_{t-k}++\sum_{k=0}^{p}\eta_{2}\Delta ATF_{t-k}^{+}+\sum_{k=0}^{p}\eta_{3}\Delta ATF_{t-k}^{-}+\sum_{k=0}^{p}\eta_{4}\Delta TFC_{t-k}^{+}+\sum_{k=0}^{p}\eta_{5}\Delta TFC_{t-k}^{-}+\sum_{k=0}^{p}\eta_{6}\Delta GFIT_{t-k}+\sum_{k=0}^{p}\eta_{7}\Delta IFS_{t-k}^{+}+\sum_{k=0}^{p}\eta_{8}\Delta IFS_{t-k}^{-}+\varsigma_{1}CDAM_{t-1}+\varsigma_{2}ATF_{t-1}^{+}+\varsigma_{3}ATF_{t-1}^{-}+\varsigma_{4}TFS_{t-1}^{+}+\varsigma_{5}TFS_{t-1}^{-}+\varsigma_{6}GFIT_{t-1}+\varsigma_{7}IFS_{t-1}^{+}+\varsigma_{8}IFS_{t-1}^{-}+\mu_{t}$$

The short-term dynamics between the variables may be determined by comparing the upper limit I(1) critical values with the Narayan critical values. After the NARDL estimates have been estimated and analyzed, they are employed as parameters in a variance decomposition analysis (VDA) to assess the long-term association between the variables.

## 4 Results and discussion

Table 1 shows the descriptive statistics of the variables. The minimum value of carbon damages is 2.852% of GNI and the maximum value of 9.097%, with an average of 5.382%. The air transportation freight has a mean value of 6983.779 million ton-km. The transportation fuel combustion reached a maximum of 8.598%, with an average value of 6.894%. The average value of greenfield investment in transportation and insurance & financial services are US$2.96E+09 and 5.819% of service imports, respectively. The trend analysis is helpful to understand the country's profile of the stated variables over a while.

**Table 1:** Descriptive statistics.

Methods	CDAM	ATF	TFC	GFIT	IFS
Mean	5.382461	6983.779	6.894754	2.96E+09	5.819505
Maximum	9.097046	25394.59	8.598695	2.60E+10	16.94228
Minimum	2.852583	46.20000	4.876900	1.73E+08	1.031658
Std. Dev.	1.772855	8380.300	1.253371	5.24E+09	2.908834
Skewness	0.363419	1.024299	0.135462	3.175920	1.259834
Kurtosis	2.165643	2.615160	1.461998	13.18314	5.871179

Note: CDAM shows carbon damages, ATF shows air transport freight, TFC shows total fuel combustion from transport, GFIT shows greenfield investment in transportation and IFS shows insurance and financial services.

Table 2 shows the correlation matrix and found that air transportation freight, fuel combustion, and greenfield investment negatively correlated with carbon damages. In contrast, insurance services have a positive correlation, although insignificant. Further, an increase in transportation fuel combustions and greenfield investment increases air cargo operations, whereas insurance services are negatively correlated, with a small correlation coefficient value. The private investment in the transportation sector increases transportation fuel combustions, which need to be replaced by green energy sources. The correlation results are not clear enough to make green transportation policies; hence, it is crucial to understand the asymmetric relationship between the variables to get some conclusive remarks on the subject matter.

**Table 2:** Correlation matrix.

Variables	CDAM	ATF	TFC	GFIT	IFS
CDAM	1				
	–				
ATF	−0.672086	1			
	(0.0000)	–			
TFC	−0.679622	0.805291	1		
	(0.0000)	(0.0000)	–		
GFIT	−0.377678	0.658715	0.494548	1	
	(0.0097)	(0.0000)	(0.0005)	–	
IFS	0.081149	−0.030254	0.022924	−0.177460	1
	(0.5919)	(0.8418)	(0.8798)	(0.2381)	–

Note: Small bracket shows probability value.

The research first used ADF and breakpoint unit root tests to determine the predicted break dates of the variables and the probable sequence of integration of the individual variables before employing asymmetric cointegration methods to comprehend the potential structural shocks presented in the model. The stated results of the unit root testing are shown in Table 3.

**Table 3:** ADF and breakpoint unit root test.

Variables	Level	First Difference	Breakpoint Unit Root Test	Level	First Difference	Decision
	Constant and Trend	Constant and Trend	Break Dates	Constant and Trend	Constant and Trend	
CDAM	−2.493 (0.328)	−5.316 (0.000)	1993 (L) 1991 (D)	−2.875 (0.942)	−6.013 (p < 0.01)	I(1)
ATF	−0.878 (0.949)	−6.930 (0.000)	2014 (L) 2001 (D)	−2.395 (0.989)	−7.142 (p < 0.01)	I(1)
TFC	−2.729 (0.230)	−6.743 (0.000)	1999 (L) 2000 (D)	−5.663 (p < 0.01)	−10.030 (p < 0.01)	I(0)
GFIT	−6.826 (0.000)	−6.141 (0.000)	2016 (L) 2010 (D)	−10.864 (p < 0.01)	−7.026 (p < 0.01)	I(0)
IFS	−4.150 (0.010)	−8.406 (0.000)	2014 (L) 1995 (D)	−6.409 (p < 0.01)	−10.626 (p < 0.01)	I(0)

Note: Small bracket shows probability value.

The results show that carbon damages and air transportation freight are differenced stationary variables with break dates of 1991 and 2001, respectively. The year 1991 was the period where carbon damages begin to rise from 8.553% of GNI. On the other hand, in 2001, air transportation freight was reached up to 4232 million ton-km. The transportation fuel combustions, greenfield transportation investment, and insurance & financial services are level stationary variables with break dates of 1999, 2016, and 2014, respectively. The stated break dates showing the following observations that linked it to some structural changes that exist in the given years, i.e., the TFC value at 1999 was 6.151% of fuel combustions, the GFIT value was US$3.47E+09 and 6.325% of service imports. Based on the different order of integration, the best option is to estimate the multivariate variables in the ARDL-Bounds testing approach, which help to give short- and long-run parameter estimates of the given variables. Before using the ARDL technique, the study checked whether the variables have an asymmetric/symmetric relationship with the response variable. Table 4 shows the short- and long term asymmetric/symmetric estimates for ready reference.

**Table 4:** Long- and short-term symmetry/asymmetry estimates.

Variables	Test Statistics	F-statistics	Probability	Conclusion
ATF	W_LR_	12.825	0.001	Asymmetric
	W_SR_	0.061	0.805	Symmetric
TFC	W_LR_	11.941	0.001	Asymmetric
	W_SR_	0.629	0.432	Symmetric
GFIT	W_LR_	2.321	0.136	Symmetric
	W_SR_	0.114	0.737	Symmetric
IFS	W_LR_	3.336	0.076	Asymmetric
	W_SR_	0.338	0.564	Symmetric

Note: W_LR_ and W_SR_ show Wald long- and short run. ATF shows air transport freight, TFC shows total fuel combustion from transport, GFIT shows greenfield investment in transportation, and IFS shows insurance and financial services.

The estimates show the asymmetric relationship between ATF, TFC, and IFS variables in response to influence on the carbon damages, which is mainly evident in the long run. Further, the variable GFIT does not show an asymmetric relationship with the carbon damages; hence its short- and long-term estimates confirmed the symmetric relationship with the response variable. The variables, i.e., ATF, TFC, and IFS, show the symmetric relationship with the carbon damages in the short run. Hence, it is evident that asymmetric causation is mainly the long-run phenomenon; hence, the study used the NARDL Bounds estimation technique to observe positive and negative shocks in the ATF, TFC, and IFS on the outcome variable. Fig. 3 shows the asymmetry plots of IFS, TFC, and IFC at a 5% confidence interval based on the estimates.

**Fig. 3:** Asymmetric plots.

Source: Author's illustration.

The estimates show that the positive shocks of IFS causing a negative impact on carbon damages, whereas the negative shocks are causing a positive impact. Thus, the given asymmetry plots fall in the 5% confidence interval that confirmed the volatility in the estimates is non-linear. Further, the positive and negative shocks in TFC on carbon damages is positive. The asymmetry pots of TFC are significant at a 5% confidence interval; hence, the non-linearity in the TFC factor is visible in the given model. Finally, the positive and negative shocks in IFS negatively impact carbon damages, which pass out through a certain threshold level. After confirming the asymmetric relationships, the study test out the cointegration bonds in five cointegrating models (see Table 5).

**Table 5:** Estimated result of ARDL bounds test.

Models	ARDL Lag length	F-statistics	Diagnostic Tests		
			J.B Test	Heteroskedasticity	LM-2 serial correlation
ln(CDAM)=f[ln(ATF),ln(TFC),ln(GFIT),ln(IFS)]	4,4,3,4,2	6.892*	4.036	1.503	2.173
ln(ATF)=f[ln(CDAM),ln(TFC),ln(GFIT),ln(IFS)]	4,3,0,1,4	2.377	5.704***	1.172	2.286
ln(TFC)=f[ln(CDAM),ln(ATF),ln(GFIT),ln(IFS)]	1,1,4,0,4	7.051*	2.239	1.091	0.622
ln(GFIT)=f[ln(CDAM),ln(ATF),ln(TFC),ln(IFS)]	1,0,0,0,0	5.476*	0.553	1.585	0.715
ln(IFS)=f[ln(CDAM),ln(ATF),ln(TFC),ln(GFIT)]	4,4,4,0,1	1.218	0.210	4.083*	1.248
**Level of Significance**	**Lower Bounds I(0)**		**Upper Bounds I(1)**		
1%	3.74		5.06		
5%	2.86		4.01		
10%	2.45		3.52		

Note: *and *** shows 1% and 10% significance level.

The estimates show that CDAM, TFC, and GFIT models are connected with their variables in the long run. The significant Wald F-statistics values fall in the upper bound (I) values; hence, any model can use in the analysis for robust inferences. The stated three models confirm with the diagnostic testing. It verified there is no normality, autocorrelation, and heteroskedasticity issue. Hence, we relied on the stated models for estimations. Before applying the NARDL technique, Table 6 shows the lag order criteria for estimation.

**Table 6:** VAR lag length criteria.

Lag	LogL	LR	FPE	AIC	SC	HQ
0	−2072.571	–	1.47e+33	99.07482	99.40580	99.19614
1	−1744.591	515.3977	5.40e+27	86.50433	89.48319	87.59620
2	−1668.730	90.31006	4.31e+27	85.93954	91.56628	88.00196
3	−1485.632	148.2224*	4.26e+25*	80.26820*	88.54281*	83.30117*

Note: * indicates lag order selected by the criterion.

The estimates show that lag up to three levels would likely give sound inferences. All of the stated lag criteria confirmed the significance of the third lag length order of the variables to get reliable estimates. Table 7 shows the NARDL estimates and found that the positive shocks in ATF negatively impact carbon damages. On the other hand, the negative shocks of ATF positively impact carbon damages in the short- and long run. The result implies that the negative shocks of air cargo operations increase more carbon damages; hence it is essential to make cargo operations green and clean. Bartle et al. [64] stressed the need to improve air freight transportation through a public-private partnership, reduction in airline schedules, improving efficiency and environmental sustainability, and green energy sources. Abrantes et al. [65] concluded that the latest technologies in aircraft could mitigate carbon emissions up to 15%. Further, shifting kerosene fuel combustions with aviation biofuels is likely to achieve green transportation agenda by attaining carbon neutrality growth.

**Table 7:** NARDL estimates.

Dependent Variable: CDAM				
Selected Model: ARDL(2, 1, 0, 3, 2, 3, 3, 2)				
Variables	Coefficient	Std. Error	t-Statistic	Prob.
D(CDAM(-1))	0.254949	0.179377	1.421300	0.1733
D(ATF_POS)	−0.000252	0.000078	−3.241662	0.0048
D(ATF_NEG)	0.000674	0.000282	2.395579	0.0284
D(TFC_POS)	0.684534	0.365722	1.871733	0.0786
D(TFC_POS(-1))	0.129968	0.246080	0.528154	0.6042
D(TFC_POS(-2))	−0.305112	0.172583	−1.767911	0.0950
D(TFC_NEG)	−1.809869	0.855088	−2.116587	0.0493
D(TFC_NEG(-1))	−1.164689	0.509768	−2.284744	0.0354
D(GFIT)	−0.000000	0.000000	−1.830714	0.0847
D(GFIT(-1))	0.000000	0.000000	1.022303	0.3210
D(GFIT(-2))	0.000000	0.000000	2.171005	0.0444
D(IFS_POS)	−0.113314	0.049406	−2.293520	0.0348
D(IFS_POS(-1))	−0.140918	0.102916	−1.369250	0.1887
D(IFS_POS(-2))	0.607475	0.202561	2.998978	0.0081
D(IFS_NEG)	0.097773	0.050573	1.933291	0.0700
D(IFS_NEG(-1))	0.193481	0.073745	2.623639	0.0178
D(@TREND(.))	0.349384	0.108695	3.214351	0.0051
CointEq(-1)	−0.908540	0.202552	−4.485458	0.0003
**Long Run Coefficients**				
ATF_POS	−0.000375	0.000050	−7.535217	0.0000
ATF_NEG	0.000742	0.000305	2.433995	0.0263
TFC_POS	1.132747	0.595745	1.901395	0.0743
TFC_NEG	−0.678168	0.731339	−0.927296	0.3668
GFIT	−0.000000	0.000000	−2.418846	0.0271
IFS_POS	−0.740110	0.243691	−3.037090	0.0074
IFS_NEG	−0.248203	0.116638	−2.127973	0.0483
C	2.199484	0.383267	5.738783	0.0000
@TREND	0.384555	0.070387	5.463403	0.0000
**NARDL Bounds Estimates**				
F-statistics	4.047	Prob.	0.040	

Further, the positive shocks of transportation fuel combustions increase carbon damages in the short- and long run. In contrast, the negative shocks of the stated variable decrease carbon damages only in the short run. Hence, the positive shocks are more prominent in the pollution damage function. It is desirable to use renewable energy sources to replace conventional gasoline and other petroleum-based fuels in cargo operations. Baxter [66] stressed the need to utilize renewable energy resources as aviation biofuels to mitigate adverse environmental externalities. Aviation biofuels help to reduce 10% to 15% GHG emissions. Hence, the feasibility of using aviation biofuels is helpful to moving towards sustainable goals. Anderson et al. [67] found that gas turbine engines in mixing fuel helpful to lower the use of fossil fuels, which reduced different pollutants combination in the atmosphere. Ng et al. [68] concluded that waste and residue feedstock could be used to produce bio-jet fuel to achieve green agenda. The greenfield investment in the transportation sector played an important role in mitigating carbon pollution and reducing carbon damages. The relationship between the stated factors is negative, confirming the viability of the private investment in transportation in making a green transportation agenda. Nieuwenhuijsen [69] suggested that sustainable transport planning and urban designing are essential for reducing transportation emissions' adverse effects, which can subsidize through public-private partnership investment. Anwar et al. [20] found that greenfield transportation investment and sustainable energy mix helpful to reduced transportation embodied carbon emissions that is important to the way forward towards sustainable development goals. Finally, the impact of positive and negative shocks of IFS on carbon damages is negative in the long run, which reinforced the capability of green insurance schemes and sustainable financing options to mitigate carbon losses related to transportation in a country [70,71]. The error correction term shows the convergence of the estimated model in the short run, with a high speed of adjustment towards equilibrium over a while.

Table 8 shows the estimates of diagnostic testing. It found that the carbon damage function passed through autocorrelation and heteroskedasticity related issues. Moreover, the Ramsey RESET and CUSUM test confirmed the model stability during the stated period.

**Table 8:** Diagnostic tests.

Methods	F-statistics	Probability value
LM Test	1.400	0.277
Heteroskedasticity Test	0.253	0.998
RESET Test	1.128	0.303
CUSUM Test	✓	p < 0.05

Finally, Table 9 shows the VDA estimates of carbon damages influenced by the positive and negative shocks of ATF, TFC, and IFS. Further, it is influenced by greenfield investment in a country. The results suggested that the negative shocks in the TFC would likely bring a more significant change in the innovation of carbon damages with an error variance shock of 19.904%. This followed the positive shocks of IFS and negative shocks of ATF with an estimated variance error of 6.077% and 4.374%, respectively. The positive shock in the TFC would be likely to bring a slight change in the carbon damage for the next 10-year time period. Based on the estimates, it is evident that transportation fuel combustion would likely impact more on carbon damages. Hence, it is vital to increase public-private investment, insurance premiums, and green financing schemes to improve air cargo operation in a country.

**Table 9:** VDA estimates of CDAM.

Period	S.E.	CDAM	ATF_NEG	ATF_POS	TFC_NEG	TFC_POS	GFIT	IFS_NEG	IFS_POS
1	0.499544	100	0	0	0	0	0	0	0
2	0.698123	93.41399	0.253333	0.037644	3.295186	0.181822	0.005337	1.121451	1.691232
3	0.863332	86.99581	0.423521	0.083707	7.879998	0.134961	0.091754	1.171683	3.218571
4	0.977428	82.21474	1.075573	0.065566	11.49127	0.107615	0.103542	0.915053	4.026634
5	1.051578	78.40747	1.995465	0.124661	13.84995	0.093004	0.116436	0.799260	4.613758
6	1.103868	74.89855	2.685481	0.178694	16.00679	0.092138	0.145852	0.729732	5.262766
7	1.138614	72.20142	3.231042	0.182217	17.83343	0.108719	0.149565	0.692549	5.601058
8	1.159574	70.38256	3.765781	0.191785	18.92540	0.116203	0.251254	0.668590	5.698423
9	1.171761	69.14605	4.188636	0.254376	19.52346	0.120883	0.272722	0.655975	5.837895
10	1.180487	68.13414	4.374707	0.375506	19.90426	0.142239	0.314965	0.676218	6.077962

## 5 Conclusions

Shipping products by aeroplane is seen as a practical business option. China's growing export industry has made it a magnet for the globalised globe. Due to their heavy reliance on petrol and other petroleum-based fuels, their logistical activities create significant environmental damage. Possible approaches to improving the aerodynamic performance of aircraft structures, including carbon fiber composites, may lighten aircraft structures. Low-takeoff and low-fuel aircraft emit less GHG. Aerodynamically efficient aircraft enhance fuel economy. Aerodynamic wing and fuselage designs may be needed. 3D printing and automated assembly may enhance aircraft structural manufacture. Modern monitoring systems may detect and analyze structural issues. Smart materials like shape-memory alloys and flexible structures may lead to aircraft constructions that adjust to operational conditions. Using up-to-date and extensive data from 1975 to 2020, this research investigates the primary damaging elements that amplify carbon damage through air freight operations in China. The NARDL method evaluates the effect of carbon damages caused by positive and negative shocks in air cargo operations, transportation fuel combustions, insurance coverage, and the greenfield investment component. The findings first confirm that an asymmetry in the pollution damage function exists, which can only be fixed by considering the aforementioned dynamic multiplier. The positive shocks of air freight transportation, the adverse shocks of transportation fuel burning, and the positive shocks of insurance services reduce short-term carbon damages. Whereas the positive shocks of transportation fuels and the adverse shocks of insurance services reduce carbon damages, the adverse shocks of air freight operations raise carbon damages. Carbon damage is reduced over the long term thanks to the positive and negative shocks provided by air travel and the insurance industry. Carbon damages are further exacerbated by the positive and negative shocks associated with air freight operations and transportation fuel combustion. Greenfield development reduces both immediate and future carbon costs. According to the VDA's calculations, adverse shocks associated with transportation fuel combustion have the greatest impact on carbon damages over any given period, followed by positive shocks associated with insurance services and adverse shocks associated with air freight operations. According to the study's estimates, the three most critical strategic strategies to achieve the ‘green is clean’ transportation goal are as follows:

i) Air cargo operations should follow an environmental sustainability standard. The use of gasoline and other petroleum-based fuels should replace by alternative sustainable fuels to minimize the adverse negative externalities. The multimodal transacting routes should use to minimize the long flight of air cargo operations. The transportation fuel combustions should be at environmental standards that do not exceed a certain amount of fueling in cargo operations. The logistics performance standards should be developed and follow through stringent environmental regulations for health safety. Air cargo linked remote market and integrated with the global economy to alleviate socio-economic problems. The competitiveness of air cargo is associated with its logistics operations that need to be monitor through environmental sustainability parameters. Fossil kerosene should replace by sustainable aviation fuels to achieve carbon neutrality agenda. Although green fuels are expensive compared to fossil kerosene, the advancement in cleaner technologies, like ‘power-to-liquid’ technology, help to reduce the price of green fueling.
ii) Sustainable insurance and financial services may help to promote green transportation infrastructure. The cargo insurance programs help to protect against the risk of damage and loss of supply chain items. Further, the insurance services should be extended to eco-friendly companies with minimum charge pricing and greater risk premium to mitigate environmental concerns. The provision of insurance to the more efficient air cargo carriers that investing in lowering emissions. Carbon offsets policies are likely to support the aviation cargo industry to adopt the latest cleaner technologies and enhanced quality and sustainability of logistics operations, and
iii) Greenfield investment in the transportation sector is vital to achieving carbon neutrality agenda. The private investment in the solutions to improve transportation infrastructure from shifting non-renewable aviation fuels to sustainable ones played an essential role in achieving the green transportation agenda. The private investment ensures safety, efficiency, and universal access to cargo facilities to a green and clean, resilient path. The need for sustainability reporting and stringent regulations remains to play their part to improve aviation cargo efficiency. More significant investment is needed to deployed renewable energy sources at airports to ensure sustainable cargo operations. The need of upgrading aviation infrastructure is essential for managing freight volumes. The investment in aviation cleaner technologies is helpful to halve the carbon emissions from transportation.

Even by examining air cargo operations, transportation fuel combustions, private investment in transportation, and insurance coverage, the research may have tended to other factors to carbon emissions in the air cargo sector, including technical development, government policy, and operational efficiency. The study focused on China's economy and air freight system. Results may be restricted by socioeconomic, infrastructural, and policy differences among countries. Electric or hybrid-electric cargo planes may reduce air freight carbon emissions, but further research is required. Studying such technology's possibilities, pros, and cons may help achieve ecologically responsible air freight operations. More research is required to establish whether legislative interventions and incentives have promoted sustainable air freight operations. Examining regulatory, financial, and market-based processes on carbon reduction programs might assist policymakers and industry actors. Comparative studies across countries or regions may help understand air freight operations and their environmental impacts. Analyzing the success rates of different countries' tactics, strategies, and legislation may help ensure air cargo operations' long-term survival. Airlines, airports, government agencies, and environmental organizations—all significant air freight players—should participate in future research. Future studies may continue to examine China's maritime transport sector's environmental impact and mitigating strategies. Comparing the air cargo business to sea transport helps comprehend sustainable transportation and inform policy choices and initiatives. Understanding their opinions, challenges, and potential carbon emission reduction solutions may improve collaboration and sustainability projects. The integrating global partnership is highly recommended to build a safe and resilient aviation cargo path to improve logistics operations and move toward a green transportation agenda.

## Production notes

### Author contribution statement

Weisong Wang; Khalid Zaman: Analyzed and interpreted the data; Contributed reagents, materials, analysis tools or data; Wrote the paper.

Wenjing Sun: Conceived and designed the experiments; Analyzed and interpreted the data; Wrote the paper.

Usama Awan: Conceived and designed the experiments; Contributed reagents, materials, analysis tools or data; Wrote the paper.

Abdelmohsen A. Nassani; Rima H. Binsaeed: Performed the experiments; Analyzed and interpreted the data; Contributed reagents, materials, analysis tools or data; Wrote the paper.

### Data availability statement

Data will be made available on request.

## Declaration of competing interest

The authors declare that they have no known competing financial interests or personal relationships that could have appeared to influence the work reported in this paper.
